RETRACTED

# Co-Depletion of Cathepsin B and uPAR Induces G0/G1 Arrest in Glioma via FOXO3a Mediated p27^Kip1^ Upregulation

**DOI:** 10.1371/journal.pone.0011668

**Published:** 2010-07-22

**Authors:** Sreelatha Gopinath, Rama Rao Malla, Christopher S. Gondi, Kiranmai Alapati, Daniel Fassett, Jeffrey D. Klopfenstein, Dzung H. Dinh, Meena Gujrati, Jasti S. Rao

**Affiliations:** 1 Department of Cancer Biology and Pharmacology, University of Illinois College of Medicine at Peoria, Peoria, Illinois, United States of America; 2 Department of Neurosurgery, University of Illinois College of Medicine at Peoria, Peoria, Illinois, United States of America; 3 Department of Pathology, University of Illinois College of Medicine at Peoria, Peoria, Illinois, United States of America; INSERM U1016, Institut Cochin, France

## Abstract

**Background:**

Cathepsin B and urokinase plasminogen activator receptor (uPAR) are both known to be overexpressed in gliomas. Our previous work and that of others strongly suggest a relationship between the infiltrative phenotype of glioma and the expression of cathepsin B and uPAR. Though their role in migration and adhesion are well studied the effect of these molecules on cell cycle progression has not been thoroughly examined.

**Methodology/Principal Findings:**

Cathespin B and uPAR single and bicistronic siRNA plasmids were used to downregulate these molecules in SNB19 and U251 glioma cells. FACS analysis and BrdU incorporation assay demonstrated G0/G1 arrest and decreased proliferation with the treatments, respectively. Immunoblot and immunocyto analysis demonstrated increased expression of p27^Kip1^ and its nuclear localization with the knockdown of cathepsin B and uPAR. These effects could be mediated by αVβ3/PI3K/AKT/FOXO pathway as observed by the decreased αVβ3 expression, PI3K and AKT phosphorylation accompanied by elevated FOXO3a levels. These results were further confirmed with the increased expression of p27^Kip1^ and FOXO3a when treated with Ly294002 (10 µM) and increased luciferase expression with the siRNA and Ly294002 treatments when the FOXO binding promoter region of p27^Kip1^ was used. Our treatment also reduced the expression of cyclin D1, cyclin D2, p-Rb and cyclin E while the expression of Cdk2 was unaffected. Of note, the Cdk2-cyclin E complex formation was reduced significantly.

**Conclusion/Significance:**

Our study indicates that cathepsin B and uPAR knockdown induces G0/G1 arrest by modulating the PI3K/AKT signaling pathway and further increases expression of p27^Kip1^ accompanied by the binding of FOXO3a to its promoter. Taken together, our findings provide molecular mechanism for the G0/G1 arrest induced by the downregulation of cathepsin B and uPAR in SNB19 and U251 glioma cells.

RETRACTED

## Introduction

Malignant glioma, a common tumor among the intracranial tumors, remains formidable despite aggressive surgery, radiotherapy and chemotherapy [1]. Cathepsin B and urokinase-type plasminogen activator receptor (uPAR) are both known to be overexpressed in gliomas and, as such, are attractive targets for gene therapy. During cancer cell invasion, these proteins, either individually or in combination, function to degrade the extracellular matrix, thereby facilitating metastasis. Our previous work and that of others strongly suggest a relationship between the infiltrative phenotype of glioma and the expression of cathepsin B and uPAR. Though their role in migration and adhesion are well studied [2]–[4], the effect of these molecules on cell cycle progression has not been thoroughly examined. Moreover, disruption of cell cycle control is a hallmark of cancer [5], [6]. In particular, the reduced expression of p27^Kip1^, which is a member of the Kip family of cyclin-dependent kinase (Cdk) inhibitors, has been extensively observed in human cancers, and its low levels are often associated with a worse prognosis [7], [8]. Increased susceptibility to cancer and multi-organ hyperplasia have been reported in p27^Kip1^-null mice [9]. It plays a crucial role in the control of cell proliferation by inhibiting the activities of complexes of G1 cyclins and Cdks and, as such, is an important candidate for therapeutic tumor suppression [10]. Some factors, including accelerated proteolysis, sequestration by cyclin D-Cdk complexes, and phosphorylation events that lead to nuclear export and/or retention in the cytosol, have significant roles in inhibiting the p27^Kip1^ function in various cancers [11]. Cytoplasmic translocation of p27^Kip1^ has been increasingly recognized in primary human tumors associated with poor survival whereas nuclear expression confers a more favorable outcome [12].

Another hallmark of most cancers, including glioma, is the increased activity of PI3K/AKT pathway that controls many biological functions like cell proliferation, survival, and insulin response [13]. Constitutive activation of this pathway facilitates tumor formation both by supporting S-phase entry and by conferring resistance to apoptotic signals that normally restrict uncontrolled cell growth [14], [15]. In the presence of growth factors, AKT negatively regulates FOXO proteins by phosphorylating them [16], [17], which results in their binding to 14-3-3 proteins and is followed by their nuclear export [18]. FOXO factors function as transcriptional activators and bind as monomers to the consensus DNA sequence TTGTTTAC [19], [20]. Depending on the cell system studied, forced expression or activation of FOXO factors triggers apoptotic responses or cell cycle arrest [21]. Cell cycle inhibitory effect of FOXO factor through increased transcription of p27^kip1^ has been reported in gliomas [22], [23]. Several integrins play important roles in promoting cell proliferation, migration and survival *in vitro* and *in vivo*. Both uPAR and cathepsin B are known to be associated in close proximity to αVβ3 integrins and has been implicated in their ability to initiate signaling events [24].

RETRACTED

In an attempt to elucidate the roles of cathepsin B and uPAR in cell cycle progression, we analyzed the activity of crucial regulators of the G0/G1 transition including p27^Kip1^ by downregulating cathepsin B and uPAR both individually and simultaneously in SNB19 and U251 glioma cells. Here, we show that shRNA-mediated downregulation of cathepsin B and uPAR results in G0/G1 arrest, prominent increased expression of p27^Kip1^ and inhibition of p-Rb. This increased expression of p27^Kip1^ correlates with decreased expression of p-PI3K, p-AKT, cyclin E, cyclin D1, cyclin D2 and increased expression of FOXO3a protein. We also show that increased expression of p27^Kip1^ is due to the efficient binding of FOXO3a on its promoter, which was analyzed by the luciferase expression.

## Results

### Knockdown of cathepsin B and uPAR decreases cell proliferation and induces G0/G1 arrest

To gain insight into the molecular roles of cathepsin B and uPAR, we knocked down the expression of these molecules using shRNA in SNB19 and U251 glioma cells and then analyzed the effects on cell proliferation and cell cycle. After 36 hrs of transfection, western blot analysis showed a 80±3% and 82±3% decrease in cathespin B expression in SNB19 and U251 cells, respectively when treated with pC (shRNA construct against cathepsinB). Cells treated with pU (shRNA construct against uPAR) did not show appreciable difference in cathespin B expression when compared to controls (98±2%). pCU-treated (shRNA bicistronic construct against cathepsin B and uPAR) cells showed 86–91% decreased expression of cathepsin B in both SNB19 and U251 cells (p<0.01). Similarly, uPAR expression was reduced by 75–80% in both cell lines when treated with pU. Cells treated with pC did not show any difference in expression when compared to controls (95±3%). uPAR expression in pCU-treated cells was significantly reduced by 80–91% (Fig. 1A) (p<0.01). Immunoblot analysis for GAPDH expression revealed equal loading. Cell proliferation analysis by BrdU incorporation assay showed that the depletion of cathepsin B and uPAR individually and simultaneously resulted in a significant reduction in the proliferation rates by: 37–40% (pU), 34–36% (pC) and 67–68% (pCU) in both cell lines (Fig. 1B). In contrast, untreated control and SV (scrambled vector)-transfected cells showed 100% proliferation in both cell lines. Similarly, MTT assay showed decreased number of cells with the treatments (pU: 38–40%; pC: 33–35% and pCU: 65–68%) compared to the controls (98–100%) in both the cell lines (Fig. S1A). Decreased growth suppression was associated with cell cycle arrest. As shown in Figure 1C, cell cycle analysis showed an increase in the G1 phase fraction with the treatments (pU: 58.34±2%, 66.68±2%; pC: 56.88±2%, 63.84±2%; and pCU: 72.16±1%, 78.45±2% in SNB19 and U251, respectively) and a concomitant decrease in the S phase (pU: 15.23±3%, 7.98±3%; pC: 16±2%, 8.56±1%; and pCU: 8.12±1%, 2.95±2% in SNB19 and U251 cells, respectively) and G2/M phase (pU: 26.43±1%, 25.34±1%; pC: 27.12±1%, 27.6±2%; and pCU: 19.12±1%, 18.6±2% in SNB19 and U251 cells, respectively) fractions. Negligible number of cells were present in sub G0/G1 phase, hence, the data is not included. Cell cycle analysis of untreated control and SV-transfected cells of SNB19 and U251 cells showed 40±5% in G1 phase, 15±10% in S phase and 32±5% in G2/M phase. These results demonstrate that the decrease in cell proliferation is due to the block of progression from G1 to S phase, and the effect was almost the same in both the cell lines. However, cell cycle analysis at 48 hrs of transfection showed significant increase (20–40%) in sub G0/G1 phase with the treatments compared to the controls (7–8%) and concomitant decrease in the G0/G1, S and G2/M phases indicating that the cells were entering into the apoptotic phase (Fig. S1B).

RETRACTED

**Figure 1:** RNAi-mediated depletion of cathepsin B and uPAR inhibits SNB19 and U251 cell proliferation and induces G0/G1 arrest. **A.** Western Blot analysis of cathepsin B and uPAR in SNB19 and U251 cells 36 hrs after transfection with SV, pU, pC and pCU. GAPDH was used as a loading control. Side panel shows quantitative analysis of cathepsin B and uPAR bands by densitometry. **B.** We analyzed cell proliferation 36 hrs after transfection using the BrdU incorporation assay and the percent of proliferation is represented graphically. Values are mean ± standard deviation (SD) from three different experiments (*p*<0.01). **C.** Propidium iodide-stained SNB19 and U251 cells were analyzed for DNA content using flow cytometry. The graph shows the percentage of cells in G0/G1, S and G2/M phases 36 hrs post transfection. Values are mean ± SD of three different experiments (*p<0.01, in comparison with the control).

### Cathepsin B and uPAR depletion affects the p27^Kip1^ expression and its subcellular localization

It is well known that p27^Kip1^ plays an important role in G0/G1 arrest. Hence, we checked the expression of p27^Kip1^ using RT-PCR and western blot analysis. RT-PCR and immunoblot analysis of pC- and pU-treated cell lysates showed increased expression of p27^Kip1^. The pCU-treated cells showed a further increase in p27^Kip1^ expression in both the cell lines. Untreated control and SV-treated cells showed very low expression of p27^Kip1^ (Fig. 2A &B). The p27^Kip1^ protein is generally phosphorylated at Ser10 and Thr187 positions and its activity depends on its phosphorylation status. Therefore, we checked the phosphorylation status of p27^Kip1^ by immunoblot analysis and found that the treatments reduced the phosphorylation of p27^Kip1^ at Ser10 and Thr187 in both the cells lines compared to the controls. Immunoflourescence staining assay revealed that the treatments induced an increase in p27^Kip1^ localization in the nucleus when compared with control cells (Fig. 2C) and a higher number of cells expressing p27^Kip1^ in the nuclei was observed with the pCU treatment (Fig. S2A). These results were further confirmed by immunoblot analysis for p27^Kip1^ protein in cytosolic and nuclear fractions (Fig. S2B).

RETRACTED

**Figure 2:** Depletion of cathepsin B and uPAR increases p27^Kip1^ nuclear localization. **A.** Expression of p27^Kip1^ and p-p27 (Ser10 and Thr187) were studied using immunoblot analysis. GAPDH was used as loading control. **B.** Total RNA isolated from untreated and treated SNB19 and U251 cells was subjected to semi-quantitative RT-PCR analysis using p27^Kip1^ primers. Data represents average of triplicates normalized to GAPDH (**p<0.01). **C.** 36 hrs after transfection with SV, pU, pC and pCU, cells were fixed, immunostained with anti-p27 antibody followed by Texas Red-conjugated anti-mouse secondary antibody. DAPI was used for nuclear staining. Representative images of three independent experiments are shown. **D.** SNB19 and U251 cells were transfected with siRNA against p27 (p27si) individually and in combination with pU, pC and pCU. The cells were also transfected with control siRNA (C-si) and SV. Thirty six hours post-transfection, cells were lysed and the total lysates were immunoblotted for p27^Kip1^, p-p27 (Ser10), and p-p27 (Thr187). **E.** Effect of the above stated treatments on proliferation was assessed using BrdU incorporation assay. The graph represents the percent of proliferating cells and the data represented are the average of three separate experiments (*p<0.05, **p<0.01, in comparison with the control).

To further confirm the role of p27^Kip1^ in growth arrest induced by the depletion of cathepsin B and uPAR, we knocked down the expression of p27^Kip1^ alone or in combination with uPAR and/or cathepsin B, and we analyzed cell proliferation using BrdU incorporation assay. As expected, immunoblot analysis showed efficient knockdown of p27^Kip1^ in p27^Kip1^ siRNA-treated cells lysates (Fig. 2D). Cell proliferation was also increased (118±2%) with the p27^Kip1^ siRNA treatment in SNB19 and U251 cells as compared to controls (97–100%) (Fig. 2E). In contrast, immunoblot analysis and BrdU incorporation assay of cells from p27^Kip1^ and cathepsin B or uPAR co-depleted cells showed a decrease in p27^Kip1^ expression but the inhibitory effect induced in proliferation by pU, pC and pCU treatments (as described in Fig. 1C) was reverted partially in co-depleted cells (pU+p27si: 82±2%, 79±2%, pC+p27si: 79±1%, 77±2% pCU+p27si: 66±2%, 64±3% in SNB19 and U251 cells, respectively) (Fig. 2E). The results indicate that cooperation from other molecules of G1 phase might be needed for complete growth arrest. When FACS analysis was performed, p27^Kip1^ knockdown and the co-depletion treatments resulted in a decrease of cells in the G0/G1 phase and a concomitant increase in cells in S and G2/M phases (Fig. S2C).

RETRACTED

### G0/G1 phase regulators

Cell cycle regulators at the G0/G1 and G1/S phase transition were analyzed after the above mentioned treatments. As p27^Kip1^ is both an inhibitor and a substrate of cyclin E-Cdk2 complex [25], we analyzed the expression of these molecules using immunoblot analysis and found that the treatments decreased the expression of cyclin E whereas the expression of Cdk2 was unaffected (Fig. 3A). Similarly, expression of αV, β3, αVβ3 integrins decreased with the treatments. Further, Cdk2 was immunoprecipitated from the cell lysates of untreated and SV, pU, pC and pCU treated SNB19 and U251 cells and immunoblotted for cyclin E. The results revealed little or no expression of cyclin E in pU, pC and pCU treated cell lysates compared to control and SV transfected cells indicating that the treatments reduced the cyclinE-Cdk2 complex formation. pCU-treated cells showed significant downregulation of cyclin E as compared to pU and pC treatments. Dimerization of αVβ3 integrin was checked by immunoprecipitating the cell lysate with β3 integrin and immunoblotted for αV integrin and found that the treatments significantly reduced the dimer formation. It was further confirmed by native gel electrophoresis by using the αVβ3 antibody (Fig. 3B).

**Figure 3:** Cathepsin B and uPAR knockdown decreases Cdk2 activity and the expression of αVβ3 integrin. **A.** Cell lysates were collected from SNB19 and U251 after transfection with SV, pU, pC or pCU. Western blot analysis of 50 µg of total cell lysates was performed to check the expression of cyclin D1, cyclin D2, Cdk2, cyclin E, Rb, p-Rb, p21, αV, β3, αVβ3 and Ki67. GAPDH was used as a loading control. **B.** Total lysates from the untreated control and SV, pU, pC or pCU-transfected cells were immunoprecipitated for Cdk2 and β3 individually and then immunoblotted for cyclin E and αV, respectively. The figure also shows the expression of αVβ3 integrin on native gel.

RETRACTED

Apart from the cyclinE-Cdk2 complex formation, the treatments also decreased the expression of cyclin D1, p21, cyclin D2 and Ki67, which is an indicator of cell proliferation (Fig. 3A). We also checked for the expression of Rb and p-Rb (Ser780 and Ser249/Thr252) as p-Rb is initially catalyzed by the complexes formed by cyclin D and Cdk4 or Cdk6 and later by cyclin E-Cdk2 [26], [27]. We found that the treatments decreased the phosphorylation status of Rb but did not affect total Rb (Fig. 3A).

### Expression of p27^Kip1^ is influenced by the upregulation of FOXO3a proteins in cathepsin B and uPAR depleted cells

Since we observed p27^Kip1^ upregulation with decreased cell proliferation and G0/G1 phase arrest with the depletion of cathepsin B and uPAR, we next determined the expression of FOXO proteins, which are important transcriptional regulators of the p27^Kip1^ promoter. We also checked for the expression of PI3K and AKT molecules, which dictate the phosphorylation status of p27^Kip1^ and affect the activity of FOXO proteins. Immunoblot analysis revealed that the expression of FOXO3a increased with the treatments, especially with pCU treatment (Fig. 4A); the treatments did not affect the other FOXO forms significantly (Fig. S3A).

**Figure 4:** Cathepsin B and uPAR knockdown induces FOXO3a expression and translocation to the nucleus by inhibiting PI3K activity. **A.** After transfection, cell lysates were collected from the untreated control and SV, pU, pC or pCU-treated cells. Equal volume of total protein was blotted for the expression of PI3K, p-PI3K, AKT, p-AKT, FOXO3a, p-FOXO3a (253), and p-FOXO3a (Ser 318). **B.** SNB19 and U251 cells were treated with either DMSO or LY294002 (Ly 10 µM) for 24 hrs as mentioned in the Materials and Methods. After incubation, the total and nuclear lysates were collected and probed for the expression of p-AKT, p27^Kip1^ (Nu), FOXO3a (Nu) and lamin B (Nu). Equal loading was confirmed by the GAPDH expression in the total cell lysate. **C.** After treatments with DMSO- and LY294002- cells were fixed, stained with propidium iodide and subjected to FACS analysis to determine cell cycle status.

RETRACTED

For FOXO proteins to be active, newly synthesized FOXO3a must translocate to the nucleus, which is further influenced by its phosphorylation status. To test whether the depletion of uPAR and/or cathepsin B affected localization of the FOXO3a protein, cytosolic and nuclear fractions were immunoblotted for FOXO3a. We found that the nuclear fractions of treated cells expressed more FOXO3a protein than the controls (Fig. S2B). Further, immunoblot analysis of total cell lysates for phospho-FOXO3a revealed that phospho-FOXO3a at Ser318 was decreased significantly more than at Ser253. As expected, the same treatments decreased the expression of phospho-PI3K and phospho-AKT; the total forms were unaffected. The effect of the treatments was the same in SNB19 and U251 cells.

PI3K is a known inhibitor of FOXO proteins. Hence, we checked the effect of the PI3K inhibitor, LY294002 (10 µM) on the expression of p-AKT in the total extracts. Western blotting revealed decreased expression of p-AKT, which is an indicator of PI3K kinase activity, and increased expression of FOXO3a and p27^Kip1^ in the nuclear extracts (Fig. 4B). FACS analysis showed that the inhibitor induced G0/G1 arrest similar to that induced by the RNAi treatments (Fig. 4C). The expression of p27^Kip1^ and FOXO3a proteins were also assessed in cathepsin B and uPAR-overexpressing cells, and we found a correlation with the above mentioned results (Fig. S3B). These results indicate that the knockdown of cathespin B and uPAR in SNB19 and U251 cells induced G0/G1 arrest with the increased expression of p27^Kip1^ and FOXO3a and reduced PI3K activity.

We further analyzed the effect of upregulation of FOXO3a on p27^Kip1^ expression at the transcriptional level. After transfecting SNB19 and U251 cells with pU, pC and pCU or after treatment with Ly294002 (10 µM), a second transfection was performed with the cDNA constructs containing the luciferase reporter gene controlled by FOXO binding promoter regions of human p27^Kip1^ [−3125 to 2845 bp (pGL-Kip1-290) and −3507 to −2478 bp (pGL-Kip1-1110)] or the consensus sequence arranged as tandem repeats in triplet (pGL-Kip1-3x) or mutated sequence (pGL-Kip1-M) or with the SV as a control. The p27^Kip1^ promoter with the normal and mutant versions of the putative FOXO binding sequence and the regions used for PCR amplification are represented in Figure 5A. Expression of luciferase was increased by 2–2.5 and 3 fold in pC- and pU-transfected cells and LY294002-treated cells, respectively when pGL-Kip1-290 (Fig. 5B), pGL-Kip1-1110 (Fig. 5C) and pGL-Kip1-3x (Fig. 5D) vectors were used. In contrast, in pCU-transfected cells, the same treatment increased luciferase expression by 4–4.5 fold. Thus, increased activity of the p27 promoter expressed as luciferase expression with the promoter constructs indicate that the regulation of p27^Kip1^ protein levels by cathepsin B and uPAR could be, at least partially, explained by the regulation of its promoter activity by increased expression of FOXO3a. The levels of luciferase expression were same with all the constructs used whereas no expression was observed either in mutated sequence driven luciferase construct (Fig. 5E) or in the SV transfected controls.

RETRACTED

**Figure 5:** Regulation of p27^Kip1^ activity in cathepsin B and uPAR-depleted glioma cells occurs through FOXO3a transcription factor. **A.** Schematic representation of the p27^Kip1^ promoter with the normal and mutant versions of the putative FOXO binding site and the regions used for PCR amplification. **B–E.** SNB19 and U251 cells were initially transfected with SV, pU, pC or pCU, and treated with Ly294002 (Ly 10 µM) separately. 24 hrs after the treatments, a second transfection with the luciferase constructs was performed as described in Materials and Methods. The luciferase expression was quantified using Promega's luciferase assay kit with a Turner Luminometer and is represented graphically. The graphs show luciferase expression when pGL-Kip1-290 (**B**), pGL-Kip1-1110 (**C**), pGL-Kip1-3x (**D**), and pGL-Kip1-M luciferase constructs were used. Assessment for luciferase expression was performed at least in triplicate (*p<0.05, **p<0.01).

### Cathepsin B and uPAR shRNA suppresses intracranial tumor growth

The effect of RNAi-mediated inhibition of cathepsin B and uPAR on pre-established tumors was studied. H&E staining revealed a large spread of tumor growth in mock and SV-treated brain sections. Whereas, pre-established intracranial tumor growth was inhibited by 95% when treated with pCU (Fig. 6A). Immunohistochemical analysis of the tumor sections from control mice for cathepsin B and uPAR showed increased expression levels localized to the tumor region while the pCU-treated tumor sections revealed very little or no expression of the cathepsin B and uPAR. When probed for the expression of p27^Kip1^ and Ki67 proteins, mock and SV-treated brain sections showed very little expression of p27^Kip1^ and increased expression of Ki67. In contrast, pCU treated brain sections showed high expression of p27^Kip1^. However, pCU-treated brain sections showed very little or no expression of Ki67 as compared to the controls (Fig. 6B), indicating that cell proliferation is inhibited by these treatments through upregulation of p27^Kip1^. The effect of the pCU treatment on tumors induced by SNB19 and U251 cells was the same.

RETRACTED

**Figure 6:** *In vivo* inhibition of tumor growth. Stereotactic implantation of SNB19 and U251 (1×10^5^) tumor cells was performed and, after one week, PBS (mock), SV or pCU was injected into the brain using an Alzet mini osmotic pump. Five animals per group were used. 30 days after implantation, the animals were sacrificed, the brains were removed and fixed, and paraffin sections were prepared. **A.** Hematoxylin and eosin staining of tissue sections to visualize tumor cells and to examine tumor volumes. Bar: 20 µM (*p<0.01) **B**. Immunohistochemical analysis of cathepsin B, uPAR, Ki67 and p27^Kip1^ in paraffin embedded tissue sections. Bar: 200 µM.

## Discussion

Various reports have demonstrated that cathepsin B and uPAR levels are overexpressed during glioma progression [28]–[30]. It has been reported that β1 integrins in caveolae bind uPAR and are linked to increased secretion of pro-cathepsin B [31]. An association of cathepsin B and uPAR mediated by active K-RAS in colorectal carcinoma has also been reported [32]. We have previously shown that RNAi-mediated downregulation of cathepsin B and uPAR led to decreased invasion, induction of angiogenesis, increased caspase-mediated apoptosis, and induction of G0/G1 arrest [2], [30], [33]–[37] Data from other reports indicate that inhibition or depletion of cathepsin B prevents cells from entering and leaving the cell cycle, thereby decreasing cell proliferation [38], [39]. However, the molecular mechanisms by which cathepsin B and uPAR regulate cellular proliferation remain poorly understood. The growing body of knowledge of genetic alterations that occur in malignant gliomas has resulted in the development of targeted therapy to restore cell cycle or apoptosis defects in gliomas [22]. In the present study, we show that the co-depletion of cathepsin B and uPAR arrests cells in the G1 phase primarily through the upregulation of p27^Kip1^ and that this pathway involves the downregulation of p-PI3K, p-AKT, D-type cyclin expression, and cyclin E/Cdk2 complex formation as well as the subsequent upregulation of the FOXO3a protein and its nuclear localization.

In the present study, we have shown that pU, pC and pCU treatments reduced endogenous levels of cathepsin B and uPAR proteins in SNB19 and U251 glioma cells (Fig. 1A) with a 75–78% transformation efficiency as obtained using GFP (Fig. S4). Among the treatments, pCU reduced protein expression more than pU and pC; this same effect was seen in the other experiments. These treatments also led to G1 arrest and decreased cell proliferation. We further investigated the influence of these treatments on p27^Kip1^ expression and localization. Western blot analysis revealed that p27^Kip1^ expression increased with the treatments while its phosphorylation at Ser10 and Thr187 decreased, thereby indicating the nuclear localization of increased p27^Kip1^ protein. This was further confirmed by the immunofluorescence analysis where the treatment showed nuclear presence of p27^Kip1^. Data from many different studies emphasize the importance of p27^Kip1^ as a potent inhibitor of cell cycle in human cancers [40]. p27^Kip1^ phosphorylation at Ser10 or Thr187 facilitates the nuclear-to-cytoplasmic redistribution of p27^Kip1^ [41], [42], and this sub-cellular localization determines the activity of p27^Kip1^. Our results suggest that reduced phosphorylation of p27^Kip1^ at Ser10 and Thr187 increased p27^Kip1^ nuclear localization, but further experiments using p27^Kip1^ siRNA and that of decreased expression of cyclin D1, cyclin D2 and cyclin E with the pU, pC and pCU treatments indicate that p27^Kip1^ alone is partially responsible for cell cycle arrest and decreased Cdk2 kinase activity might be necessary to complete the task. Similar results showing that SHP1 downregulation effected p27^Kip1^ expression and Cdk2-cyclin E complex formation have been reported [43]. However, we were unable to find any translocation difference of Cdk2 with the treatments as observed by [43]. Our immunoprecipitation results indicate that Cdk2 kinase activity was reduced with the treatments. As a member of the CIP/KIP family, p27^Kip1^ was found to be associated with and to inhibit the catalytic activities of G1 and S phase-specific Cdk/cyclin complexes [44]. Thus, the decrease in p-p27^Kip1^ with the treatments could be due to the low Cdk2 kinase activity. Our results also indicate decreased phosphorylation of Rb at Ser780 and Ser249/Thr252. Inactivated retinoblastoma (p-Rb) protein regulates the progression from G1 to S phase through its association with the E2F family of transcription factors [45], [46]. In early and late G1 phase, p-Rb is hyperphosphorylated by D-type Cdks and Cdk2-cyclin E, respectively [26], [47], [48]. These reports suggest conclusively that phosphorylation of p-Rb by Cdk2-cyclin E requires p-Rb to be hypophosphorylated, and thus, the inactivation of p-Rb involves sequential phosphorylation by cyclin D-Cdk4/6 and cyclin E/Cdk2 [26], [27]. Therefore, the G0/G1 arrest induced by the treatments could be due to the combined action of reduced cyclin D1, cyclin D2, and cyclin E-Cdk2 complex formation and increased expression of p27^Kip1^.

RETRACTED

Hyperactivation of the PI3K-AKT pathway is critical in human tumorigenesis because it promotes cell growth, survival and resistance to treatment [49], [50]. In addition, it has been reported that 88% of gliomas show altered PI3K-AKT signaling [51]. Integrins on tumor cells increases tumor cell migration, invasion, proliferation and survival [52]. In this study, we have shown that downregulation of cathepsin B and uPAR significantly decreased the dimer formation of αVβ3 integrins as seen in immunoprecipitation and native gel electrophoresis with the decreased expression of both αV and β3 integrins. The roles of other integrins are being investigated in our laboratory. Transcriptional downregulation of p27^kip1^ mRNA by AKT occurs through localization and subsequent inhibition of the FOXO protein. Recent data show FOXO3a directly regulates p27^kip1^ transcription [53], [54], suggesting that reduced p27^kip1^ levels after a proliferative stimulus may also be associated with FOXO3a. Our results further confirm these findings. In the present study, FOXO3a expression was positively correlated with p27^kip1^ expression (Fig. 2A) but inversely associated with cell proliferation as identified by Ki67 (Fig. 3A), which is a marker of cell proliferation expressed specifically in the cell nucleus from late G1 to S phase. We observed a decrease in phosphorylation of PI3K, AKT and FOXO3a (Ser318) (Fig. 4A) protein along with decreased activity of Cdk2 (Fig. 3B) with the RNAi treatments. Activated AKT is crucial in preventing FOXO3a displacement to the nucleus [55], [56]. However, AKT-independent and Cdk2-dependent phosphorylation affected FOXO1 nuclear export to different extents in U87 and U251 glioma cells [22]. Our results reveal that LY294002 significantly inhibited the phosphorylation and activation of AKT. More importantly, LY294002-treatment caused FOXO3a nuclear accumulation. These results suggest that LY294002 controlled the activity of FOXO3a by regulating its phosphorylation and subcellular localization. It is known that FOXO3a regulates the transcription of p27^kip1^ by binding to its promoter [57]. Indeed, we found that p27^kip1^ expression increased with LY294002 treatment. Moreover, after treatment with pU, pC, pCU and Ly294002, luciferase expression under the influence of FOXO binding promoter region of p27^Kip1^ increased with the treatments as compared to control and SV-transfected cells. Among the treatments, pCU-treated cells showed more luciferase activity than pU- and pC-treated cells. Notably, luciferase expression was nearly the same irrespective of the vector used. Studies have indicated that other transcription factors, such as Sp1, CRE and NF-κB, regulate p27^Kip1^ promoter activity [58], [59]. Very recently, Li [60] reported the effect of anti-inflammatory drugs on proliferation of human osteoblasts with the increased activity of FOXO3a by binding to p27^Kip1^ promoter. Thus, these findings invite the conclusion that the increased p27^Kip1^ expression with the treatments is due to the increased nuclear expression of FOXO3a, which binds to the -2984 bp region on the p27^Kip1^ promoter and could be mediated by the low expression of p-AKT. The results obtained were also confirmed by immunoblotting for p-PI3K, p-AKT, FOXO3a and p27^Kip1^ in the cathepsin B and uPAR-overexpressed SNB19 and U251 cells.

RETRACTED

Although overexpression of p27^Kip1^ can induce protection from apoptosis, other studies have reported pro-apoptotic effects where caspases are able to cleave p27^Kip1^ in a cell type specific manner [9], [61] reported that the inhibition of cytochrome c release might be a possible mechanism of preventing apoptosis with higher p27^Kip1^ expression in leukemia cells; this indicates that the regulation of the apoptotic process by p27^Kip1^ might vary with cell transformation status. In a separate experiment, we observed decreased expression of p27^Kip1^ in the nucleus at the 72 hours time point (data not shown). Several recent reports have shown that p27^Kip1^ has cell cycle-independent functions, such as the regulation of cell migration, which might be oncogenic under certain circumstances [25].

The efficiency of *in vivo* RNAi/adeno virus treatments by targeting proteins like uPA and uPAR [62], cathepsin B and uPAR [3], and uPAR and MMP-9 [63] has been well established in our laboratory. Similarly, the present study demonstrates that the simultaneous downregulation of cathepsin B and uPAR caused the regression of intracranial tumors. Nude mice implanted intracranially with SNB19 and U251 glioma cells became very weak within three to four weeks due to tumor development. In contrast, pCU-treated mice were healthy, and H&E staining of these tissue sections revealed very few to no cancer cells as compared to the controls. Interestingly, we observed high expression of p27^Kip1^ and very low expression of Ki67 in the tumor sections, indicating the efficiency of treatment both *in vitro* and *in vivo*. Moreover, a direct correlation between the low expression of p27^Kip1^ and FOXO3a and higher expression of Ki67 with the malignant glioma has been reported [23]. Increased expression of p21 and regression of lung tumor growth *in vivo* with the administration of decorin has been reported [64]. Yu [65] has reported that the downregulation of uPAR induced G0/G1 arrest *in vitro* but did not affect growth *in vivo*. Decreased tumor growth and metastasis of malignant melanoma cells in nude mice with the administration of antisense oligonucleotide for uPAR has been described [66]. Likewise, an 88% inhibition of proliferating cancer cells in colorectal carcinoma *in vivo* when treated with uPAR monoclonal antibody (ATN658) has been reported recently [67]. In contrast, uPAR overexpression inhibited cell growth in murine embryonic fibroblast cells and induced cell growth in keratinocytes [68]. uPAR has been detected as a potential cooperating oncogene in Ink4a KO mice, which are deficient in cell growth control [69]. Thus, the effect of uPAR on growth rate may depend on cell type. Not much has been reported about cathepsin B controlling cell proliferation *in vivo*. In conclusion, our results demonstrate that Akt/FOXO3a/p27^Kip1^ signaling contributes to G0/G1 arrest, which was induced by the depletion of cathepsin B and uPAR (Fig. 7). Moreover, our results also demonstrate that the bicistronic construct, pCU, was more effective than the single constructs, pU and pC. Thus, our findings provide molecular mechanism for the G0/G1 arrest induced by the downregulation of cathepsin B and uPAR in SNB19 and U251 glioma cells.

RETRACTED

**Figure 7:** Schematic representation of the molecular mechanisms proposed in the regulation of cell proliferation by G0/G1 arrest with the increased expression of FOXO3a and p27^Kip1^ in cathepsin B and uPAR-depleted glioma cells.

## Materials and Methods

### Ethics Statement

The Institutional Animal Care and Use Committee of the University Of Illinois College Of Medicine at Peoria, Peoria, IL, USA approved all surgical interventions and post-operative animal care. The consent was written and approved. The approved protocol number is 851, dated November 20, 2009. No de novo cell lines were used.

### siRNA constructs, cell culture, transfection and inhibitor treatments

Single shRNA constructs directed against uPAR (pU) and cathepsin B (pC) and the bicistronic construct directed against both cathepsin B and uPAR (pCU) have been described previously [2]. siRNA for p27^Kip1^ (p27si) was purchased from Santa Cruz Biotechnology (Santa Cruz, CA). Full length cathepsin B and uPAR over expressing plasmids were purchased from Origene (Rockville, MD). All the antibodies used in this study are from Santa Cruz Biotechnology (Santa Cruz, CA) unless otherwise mentioned.

Human glioma cell lines SNB19 and U251, obtained form American Type Culture Collection (ATCC, Manassas, VA) were cultured in DMEM/high glucose media supplemented with 10% FBS in a humidified atmosphere containing 5% CO_2_ at 37°C. Cells were grown in 100 mm dishes for all treatment conditions and on two-well chamber slides for immunocytochemistry analysis. Scrambled vector (SV- sequence corresponds to the bicistronic shRNA directed against the cathepisn B and uPAR), pU, pC and pCU vectors were transfected into SNB19 and U251 cells independently with Fugene 2000 reagent as per the manufacturer's instructions (Roche, Indianapolis, IN). For the inhibitor study, cells seeded in six well plate were treated with Ly294002 (10 µM), a potent PI3K inhibitor, for 24 hrs.

RETRACTED

### Cell proliferation assay and cell cycle analysis

Cell proliferation analysis was performed using Cell Proliferation ELISA (colorimetric) BrdU incorporation assay (Roche diagnostics, Indianapolis, IN), according to the manufacturer's protocol. Cell viability analysis was performed by MTT assay using the Cell Titer 96 colorimetric assay as described previously [3]. Phases of cell cycle were analyzed using flow cytometry after 36 hrs and 48 hrs of transfection. Cells were trypsinized, washed with 1X PBS, fixed and permeabilized with cold 70% ethanol and finally incubated for 30 min with 1 mL of propidium iodide (conatins NP-40) (Biosure, CA) in the dark. The DNA content of these cells was measured based on the presence of propidium iodide (PI)-stained cells. Flow cytometric analysis was done on at least 10,000 cells from each sample, and cell cycle data were analyzed using a FACS Calibur flow cytometer (BD BioSciences, San Jose, CA) with an excitation wavelength of 488 nm and emission wavelength of 530 nm.

### RT-PCR, Western blot and immunoprecipitation analysis

36 hrs after transfection, total RNA was isolated using Trizol reagent (Invitrogen, Carlsbad, USA) and converted to cDNA using Transcriptor First Strand cDNA synthesis kit (Roche diagnostics, Indianapolis, IN) as per manufacturer's instructions. PCR was performed for p27 mRNA expression using forward 5′TCAAAGCAAGCTCTTCATACCC3′ and reverse 5′GCACATAAACTTTGGGGAAGG3′ primers. For immunoblot analysis, cells were washed with ice-cold DPBS and resuspended in 150 µL of radioimmune precipitation assay buffer. The cell lysates were analyzed by SDS-PAGE followed by western blotting. The following antibodies were used: uPAR, cathepsin B, (Athens Research and Technology, Athens, GA, USA) αV (Millipore, Billerica, MA), β3, αVβ3, PI3K, p-PI3K, AKT, p-AKT (Cell Signaling, Boston, MA), p21, p27^Kip1^, p-p27^Kip1^ (Ser10), p-p27^Kip1^ (Thr187), cyclin D1, cyclin D2, Cdk2, cyclin E, Ki67, FOXO3a, p-FOXO3a (Ser253), FOXO3a (Ser318/321), FOXO1, p-FOXO1 (Ser256) (Cell Signaling, Boston, MA), Rb, p-Rb (Ser780 and Ser249/Thr252) and GAPDH. Signals were detected using Pierce Western Blotting substrate (Pierce, Rockford, IL), and the chemiluminescent images were captured in the Flourchem Q, Alpha Innotech, Gel Documentation system. Also, a native gel electrophoresis (7%) was performed on PAGE in the absence of SDS without denaturing the proteins to check the dimerization of αVβ3 integrin

β3 and Cdk2 was immunoprecipitated from 300 µg of total protein using anti- β3 and -Cdk2 antibody and protein A plus G agarose beads (20 µg). The precipitates were washed five times with lysis buffer and once with PBS. The pellet was then resuspended in sample buffer (50 mM Tris, (pH 6.8), 100 mM bromophenol blue, and 10% glycerol) and incubated at 90°C for 10 min before electrophoresis to release the proteins from the beads and immunoblotted for αV and cyclin E, respectively.

RETRACTED

### Isolation of nuclear and cytoplasmic cell fractions

Cytoplasmic and nuclear extracts from the treated cells were isolated using Active Motif nuclear extraction kit (Active Motif, Carlsbad, CA) according to the manufacturer's instructions. Harvested cells were washed once with 1X PBS, the cell pellet was resuspended in 200 µL of hypotonic buffer, incubated for 30 min at 4°C on a rocking platform, and centrifuged. The supernatant was collected as the cytosolic fraction. The nuclear pellet was resuspended, homogenized and incubated in complete lysis buffer provided in the kit for 30 min at 4°C on a rocking platform, and the nuclear fraction was collected after centrifugation. Immunoblot analysis was performed with the cytoplasmic and nuclear fractions for proteins like p27^Kip1^ and FOXO3a. Nuclear fractions were also tested for the expression of the lamin B.

### Immunofluorescence assay

Human glioma cells (SNB19 and U251) grown in two-well chamber slides were treated as described earlier. The cells were washed with PBS, fixed with 4% paraformaldehyde, permeabilized with ice-cold methanol, and rehydrated with PBS. PBST containing 2% BSA was used for blocking the cells for one hour followed by a two-hour incubation with anti-p27^Kip1^ antibody (Cell Signaling, Boston, MA) at a dilution of 1∶300 in PBST containing 2% bovine serum albumin, followed by a final incubation with Texas Red conjugated secondary antibody (1∶1000 in PBS/2% bovine serum albumin, 0.5% tween 20) for one hour. Expression was visualized by fluorescence microscopy ((Olympus IX71; Olympus Optical Co, Tokyo, Japan)) and photographed.

### Construction of human p27^Kip1^ promoter reporter vector and luciferase activity

To determine the FOXO influenced promoter activity of p27^Kip1^, three tandem repeats of FOXO binding consensus sequence (GACTGTAAACAAAAC) comprising a 5′ end phospho modification and *Sac*I and *Xho*I restriction sites on 5′and 3′ends of upper and bottom strands, respectively, were cloned into the pGL3 basic vector and labeled as pGL-Kip-13x. The consensus sequence is positioned at −2984 to −2992 bp. Another plasmid was constructed by altering the consensus sequence (TTGTTTACAA to TTGTGCGCTA) to serve as a negative control and also to show the specificity of the consensus sequence towards FOXO. Similarly, the human p27^Kip1^ promoter was amplified from genomic DNA using the following primers:

F- aaa**GAGCTC**CCCACTTTGCAGAAGGATG and

R-aaaCTCGAGGAGCACCATTTTGTCGCTTT;

F-aaa**GAGCTC**ACCTTCGCAGAAACATTTGG and

R-aaa**CTCGAG**GCAAGAGGTCTCATCCTCTTTA with *Sac*I and *Xho*I restriction sites on 5′ and 3′ regions of forward and reverse primers, respectively. These primers amplify a 290 bp (located between −3125 to 2845 bp) and an 1110 bp (located between −3507 to −2478 bp) region that includes the FOXO binding consensus sequence. The PCR product was cloned into the promoter-less luciferase reporter vector, pGL3 basic (Promega), predigested with *Sac*I and *Xho*I, and labeled as pGL-Kip1-290 and pGL-Kip1-1110, respectively.

RETRACTED

Luciferase activity was measured with Promega's luciferase assay kit. Following 24 and 48 hrs of transfection, cells were washed twice with PBS and lysed with 100 mL of reporter lysis buffer. The lysate was shaken at room temperature for 10±15 min, after which 20 µL of each cell lysate was mixed with 100 µL of buffer and measured for luciferase activity in a Turner Luminometer (Turner Designs, Sunnyvale, CA, USA) over an integration period of 15 sec. Values obtained were normalized to GAPDH levels.

### Intracranial glioma cell implantation, treatment and immunohistochemistry

Stereotactic implantation of SNB19 and U251 glioma cells (1×10^5^), followed by treatments with mock, SV and pCU using Alzet minipumps at the rate of 0.25 µL/hr, the eventual sacrifice of glioma-bearing mice, and tumor processing were carried out as previously described [62], [70]. Sections were stained with hematoxylin and eosin (H&E) to visualize tumor cells and to examine tumor volume as described earlier [3], [71]. The sections were evaluated by a neuropathologist who was blinded as to the treatment group and scored semiquantitatively for tumor size, as described previously [3], [71]. Five animals were used per treatment. The average tumor area per section integrated to the number of sections where the tumor was visible was used to calculate tumor volume and compared between controls and treated groups. Immunohistochemistry for p27^Kip1^, cathepsin B, uPAR and Ki67 was performed as described earlier.

### Statistical analysis

Values are shown as means ± SD of at least three independent experiments. Results were analysed using a two-tailed Student's t-test to assess statistical significance. p<0.05 was considered significant.

## Supporting Information

Figure S1 RNAi-mediated depletion of cathepsin B and uPAR affects cell viability and proliferation in SNB19 and U251. A. We analyzed cell viability 36 hrs after transfection using the MTT assay, and the percent of viable cells are represented graphically. Values are mean ± standard deviation (SD) from three different experiments (p<0.01). B. After 48 hrs of transfection with SV, pC, pU and pCU, cells were collected, stained with propidium iodide and analysed for DNA content using flow cytometry. The graph shows the percentage of cells in sub G0/G1, G0/G1, S and G2/M phases. Values are mean ± SD of three different experiments (*p<0.01).
(0.14 MB TIF)

Figure S2 Cathepsin B and uPAR knockdown induces p27^Kip1^ and FOXO3a nuclear translocation. A. The ratio of nuclear vs cytoplasmic distribution of p27^Kip1^ in SNB19 and U251 cells after immunocyto analysis for p27^Kip1^ were calculated and represented graphically. The values are an average calculated from ten different fields (*p<0.01). B. After transfection with SV, pU, pC and pCU, SNB19 and U251 cells were collected, and proteins from the cytosolic and nuclear fractions were isolated. Immunoblot analysis was performed for the expression of p27^Kip1^ and FOXO3a in nuclear fractions. The RNAi treatments increased the expression of the above mentioned molecules. C. Glioma cells were treated with siRNA for p27^Kip1^ individually and in combination with SV, pU, pC and pCU. The cells were subjected to FACS analysis. The graph shows the percent of cells distributed in G0/G1, S and G2/M phases of cell cycle. Values are mean ± standard deviation (SD) from three different experiments (*p<0.01).
(5.63 MB TIF)

Figure S3 FOXO1 expression is unaffected by treatment with pU, pC and pCU; p27^Kip1^ and FOXO3a expression decreases with the upregulation of cathepsin B and uPAR. A. Immunoblot analysis of total protein isolated from transfected SNB19 and U251 cells. Immunoblot analysis was performed for the expression of FOXO1, p-FOXO1 (Thr24), p-FOXO1 (Ser256), p-FOXO1 (Ser319)/FOXO4 (Ser262), p-FOXO4 (Ser262) and GAPDH. B. SNB19 and U251 cells were transfected either with SV or full length uPAR (fl-U) or full length cathepsin B (fl-C). Total cell lysates were collected and immunobloted for the expression of uPAR, cathepsin B, p-PI3K, p-AKT, p27^Kip1^, FOXO3a and GAPDH.
(0.62 MB TIF)

Figure S4 Transfection efficiency in glioma cells. Glioma cells were transfected with GFP using Fugene (1∶3, Fugene: plasmid ratio). Shown are the images, after transfections,taken under bright and fluorescent fields.
(0.46 MB TIF)
